# Identification of Potential Therapeutic Target Genes in Osteoarthritis

**DOI:** 10.1155/2022/8027987

**Published:** 2022-08-13

**Authors:** Yang Hu, Yinteng Wu, Fu Gan, Mingyang Jiang, Dongxu Chen, Mingjing Xie, Yiji Jike, Zhandong Bo

**Affiliations:** ^1^Department of Orthopedics, The First Affiliated Hospital of Guangxi Medical University, Nanning 530021, China; ^2^Department of Urology Surgery, The Affiliated Hospital of Youjiang Medical University for Nationalities, Baise 533000, China; ^3^Department of Joint Surgery and Sports Medicine, Nanxishan Hospital of Guangxi Zhuang Autonomous Region, Guilin 541002, China

## Abstract

**Objective:**

Osteoarthritis (OA), also known as joint failure, is characterized by joint pain and, in severe cases, can lead to loss of joint function in patients. Immune-related genes and immune cell infiltration play a crucial role in OA development. We used bioinformatics approaches to detect potential diagnostic markers and available drugs for OA while initially exploring the immune mechanisms of OA.

**Methods:**

The training set GSE55235 and validation set GSE51588 and GSE55457 were obtained from the Gene Expression Omnibus (GEO) database and differentially expressed genes (DEGs) were identified by the limma package. Gene set enrichment analysis (GSEA) was performed on the GSE55235 dataset using the cluster profiler package. At the same time, DEGs were analyzed by gene ontology (GO) and the Kyoto Encyclopedia of Genes and Genomes (KEGG). In addition, protein-protein interaction (PPI) analysis was performed on the common DEGs of the three datasets using the STRING database. Proteins with direct linkage were identified as hub genes, and the relation of hub genes was subsequently analyzed using the GOSemSim package. Hub genes' expression profiles and diagnostic capabilities (ROC curves) were analyzed and validated using three datasets. In addition, we performed RT-qPCR to validate the levels of hub genes. The immune microenvironment was analyzed using the CIBERSORT package, and the relationship between hub genes and immune cells was evaluated. In addition, we used a linkage map (CMAP) database to identify available drug candidates. Finally, the GSEA of hub genes was used to decipher the potential pathways corresponding to hub genes.

**Results:**

Three hub genes (*CX3CR1*, *MYC*, and *TLR7*) were identified. *CX3CR1* and *TLR7* were highly expressed in patients with OA, whereas the expression of *MYC* was low. The results of RT-qPCR validation were consistent with those obtained using datasets. Among these genes, *CX3CR1* and *TLR7* can be used as diagnostic markers. It was found that CX3CR1, MYC, and TLR7 affect the immune microenvironment of OA via different immune cells. In addition, we identified a potential drug for the treatment of OA. Altogether, CX3CR1, MYC, and TLR7 affect the immune response of OA through multiple pathways.

**Conclusion:**

CX3CR1, MYC, and TLR7 are associated with various immune cells and are the potential diagnostic markers and therapeutic targets for OA.

## 1. Background

Osteoarthritis (OA) refers to a common arthritic disease worldwide, featured by several changes such as synovial inflammation, cartilage degeneration, and subchondral bone sclerosis [1]. It affected more than 500 million people worldwide (∼7% of the global population), with exceptionally high prevalence in those of advanced age (>65 years of age) [2]. Factors contributing to OA include joint trauma, age, obesity, joint shape, and alignment [3]. However, recently, more and more research has demonstrated the crucial function of immune molecules in the pathogenesis of OA, such that OA is gradually recognized as a chronic inflammatory response [4]. At present, OA is routinely diagnosed according to clinical presentations and a combination of imaging technologies [5]. Unfortunately, an early, accurate OA diagnosis remains impossible, and there exists no effective drug for its treatment. Therefore, it is highly crucial to explore early diagnostic biomarkers that can also serve as drug targets to enhance the prognosis and treatment of patients undergoing OA.

Due to the development of bioinformatics technology, high-throughput platform-based gene chips have emerged as an effective tool to study gene expression profiles and explore molecular mechanisms underlying several diseases [6]. This approach is considered an efficient method for identifying diagnostic markers and therapeutic targets. CIBERSORT, an algorithm used to depict the immune cell constitution within complicated tissues using the corresponding gene expression patterns, is extensively adopted for assessing the relative abundances of 22 immune cells in multiple diseases [7]. Thus, it can be applied for analyzing infiltration degrees of immune cells within OA, which can thus facilitate to development of novel diagnostic biomarkers and immunotherapeutic targets.

We first downloaded three OA microarray datasets in Gene Expression Omnibus (GEO) database, and differentially expressed genes (DEGs) were analyzed. Afterward, the common DEGs in the two datasets were used for protein-protein interaction (PPI) studies for selecting and determining diagnostic markers for OA. In addition, this study identified drugs that acted on the product of these genes. We used CIBERSORT to explore the differences in immune infiltration degrees within OA compared with healthy tissue samples of 22 immune cell types. Apart from that, this work also investigated the association of diagnostic markers with infiltration degrees of immune cells. Finally, a single-gene Gene Set Enrichment Analysis (GSEA) was conducted to identify immune pathways related to diagnostic markers to better understand molecular immune mechanisms related to OA occurrence and progression.

## 2. Methods

### 2.1. Data Collection

To identify genome-wide gene expression datasets comparing gene expression in OA tissues and normal tissues, we searched and selected the GSE55235, GSE51588, and GSE55457 datasets for subsequent analysis using the Gene Expression Overview (GEO) database. We used GSE55235 as the training set, whereas GSE51588 and GSE55457 as validation sets.

### 2.2. Screening of Differentially Expressed Genes

Using the information obtained from the GPL96 platform, the probe identification number was first converted to a traditional gene symbol, and the maximum value was assigned to multiple probes of the same gene as the gene expression. Datasets were normalized and differentially expressed using the limma software package. The criteria for screening DEGs were adjusted *P* < 0.05 after correction; |log FC|> 1.5, FC refers to the fold of difference.

### 2.3. Gene Set Enrichment Analysis

GSEA detects changes in expression in the sets of genes rather than individual genes. Therefore, subtle changes in the expression can be found, and better results can be obtained. To identify the biological processes and GO terms, together with KEGG pathways associated with OA, we performed GSEA on the GSE51588 dataset with cluster profiler *R* package, with *P* < 0.05 indicating statistical significance.

### 2.4. Functional Annotation of DEGs

Gene Ontology (GO) is classified into three types, namely, biological process (BP), cellular component (CC), and molecular function (MF). It is a broad and highly efficient method to interpret gene products and their functional characteristics. The KEGG analysis provides a data resource about known metabolic pathways to understand higher-level functions of genes and biological systems. As a package for annotation, visualization, and integrated discovery, a cluster profiler can be adopted for extracting meaningful biological information about genes. DEGs from the training set were examined with a cluster profiler software package, and a *P* < 0.05 threshold was considered significant.

### 2.5. Protein-Protein Interaction Network (PPI and Hub Gene Selection)

We extracted DEGs from the GSE55235 dataset and intersected them with those from GSE51588 and GSE55457 datasets, respectively, to obtain the common DEGs between the two datasets. The online tool VennDetail was used to construct the common DEGs between two datasets, respectively. STRING database (https://string-db.org) was adopted to retrieve interacting genes/proteins, including approximately 24.6 million proteins and over 3.1 billion interactions in 5.09 K organisms. In the STRING database, we selected “multiple proteins,” entered co-up-and down-regulated differential genes, selected “*Homo sapiens*” as the organism, and set the significant threshold to the lowest interaction score >0.4 (low confidence). Subsequently, the Cytoscape software the PPI network was constructed using. We analyzed the key genes using the GOSemSim package to analyze their functional similarity. This analysis was based on the assumption that if two gene products are functionally similar, they tend to be located together in the GOtree.

### 2.6. Expression-Level Validation of Hub Genes

The genes in the GSE55235 dataset were extracted, and their expression was analyzed and verified using the GSE51588 and GSE55457 datasets.

### 2.7. Experimental Validation of Hub Gene Expression

We obtained rat articular chondrocytes from Wuhan Procell Life Science and Technology Co., Ltd. Cells were cultured using DMEM/F12 medium containing 10% fetal bovine serum. The inflammation model group was stimulated with a medium containing IL-1*β* at a concentration of 10 ng/ml for 24 h. Total RNA was extracted with RNAeasy™ Animal RNA Extraction Kit (Beyotime Biotechnology, China), and quality control was conducted by NanoDrop one spectrophotometer. Then, reverse transcription was performed to produce cDNA. The extracted RNA was reverse transcribed to cDNA using PrimeScript™ RT Master Mix (TAKARA, Japan). cDNA was extracted using PowerUp™ SYBR® Green Master Mix (Applied Biosystems, USA) and ABI 7500Real-TimePCR System. RT-qPCR was performed to detect the expression of differential genes. GAPDH was used as an internal reference. The relative mRNA expression level was calculated with the 2^−ΔΔCt^ method, and *P* < 0.05 indicated a significant difference. The primer sequences are shown in Table 1.

### 2.8. ROC-Level Validation of Hub Genes

In the GSE55235 database, the total RNA was extracted from patients undergoing OA and healthy controls. The ROC curves were drawn. At the same time, the area under the curve (AUC) was computed using “proc” software to evaluate the ability of the selected genes, aiming to discriminate between patients with OA and controls. Both GSE51588 and GSE55457 datasets were used to validate their ROC levels.

### 2.9. Correlation Analysis of Hub Gene with Immune Cells

This work employed *R* package CiberSort to process the GSE55235 gene expression matrix data. Besides, samples satisfying *P* < 0.05 were chosen for obtaining the infiltration matrix of OA immune cells. For visualizing the proportions of 22 immune cell infiltrations within patients with OA, the cumulative histogram was plotted using the “ggplot2” software package. Correlations between 22 immune cells were analyzed and visualized using the “corrplot” software package. This study drew violin plots with “ggplot2” package for visualizing different infiltration degrees of immune cells in OA compared with normal groups.

### 2.10. Correlation Analysis of Hub Gene with Infiltration Degrees of Immune Cells

This work conducted Spearman's correlation on immune cells and hub genes, and immune cells satisfying *P* < 0.05 were chosen. The ggplot2 software package was used to visualize the results.

### 2.11. Small Molecule Drug Analysis

As an experimentally validated drug database, the CMAP database can be used to predict the potential molecular compounds acting on OA. CX3CR1, MYC, and TLR7 were submitted to the CMAP website to identify small-molecule drugs against OA. The correlation between the drug and the target is represented by a score of −1 to 1, with negative scores indicating that the drug has the potential to inhibit OA. Therefore, enrichment <0 and *P* < 0.001 were used for screening.

### 2.12. GSEA of Hub Genes

To further explore the potential functions of CX3CR1, MYC, and TLR7 in OA, GSEA was performed on CX3CR1, MYC, and TLR7. In the GSE51588 dataset, according to the expression of CX3CR1, MYC, and TLR7, Spearman's analysis was used to calculate their correlation coefficients with other genes. They were treated as an ordered gene list. The R package “cluster profile” was used to select hall.v7.4.sytmbols.gmt from the Molecular Signature Database (MSigDB) as the reference genome for GSEA, and a *P* -adjustment value < 0.05 was used as the screening criterion.

## 3. Results

### 3.1. Screening Results of DEGs

The limma software package analysis revealed 343 standard-compliant DEGs from the GSE55235 dataset, among which 167 showed up-regulation while 176 showed down-regulation (Figure 1(a)). In the GSE51588 dataset, 272 standard DEGs were discovered, including 108 with up-regulation, replaced by 164 with down-regulation (Figure 1(b)). In addition, we discovered 109 qualified DEGs from the GSE55457 dataset, including 26 with up-regulation and 83 with down-regulation (Figure 1(c)). The respective top 15 up-regulated and down-regulated genes in the GSE55235, GSE51588, and GSE55457 datasets are shown in the heatmap (Figures 1(d) and 1(f)).

### 3.2. GSEA

Gene set enrichment analysis revealed that compared with controls, the gastrointestinal system's smooth muscle contraction, glycosphingolipid catabolic process, response to UV-A, and glycolipid catabolic processes were enriched in BP (Figure 2(a)). The major histocompatibility complex (MHC) class II protein complex, immunoglobulin complex, banded collagen fibrils, and fibrillar collagen trimer were enriched in CC (Figure 2(b)). In MF, platelet-derived growth factor binding, immunoglobulin receptor binding, peptidoglycan binding, and immunoglobulin binding were mainly enriched (Figure 2(c)). The KEGG analysis revealed enrichment in asthma, autoimmune thyroid disease, N primary immunodeficiency as well as intestinal immune network for IgA production (Figure 2(d)).

### 3.3. DEGs Functional Enrichment Analysis Results

GO as well as KEGG enrichment analysis was conducted with the cluster profiler package in R for exploring DEGs' biological functions. In the BP group, we enriched DEGs in neutrophil degranulation, neutrophil activation, as well as neutrophil activation involved in immune response (Figure 3(a)). In the CC group, DEGs were majorly concentrated in secretory granule lumen, vesicle lumen, and cytoplasmic vesicle lumen (Figure 3(b)). In the MF group, DEGs were associated with glycosaminoglycan binding, extracellular matrix structural constituents, and heparin-binding (Figure 3(c)). In KEGG, DEGs were enriched in neutrophil extracellular trap formation, viral protein interaction with cytokines or their receptors, and *Staphylococcus aureus* infection (Figure 3(d)).

### 3.4. PPI Network Construction and Key Gene Screening

Two up-regulated DEGs (*CX3CR1* and *TLR7*) and two down-regulated DEGs (*MYC* and *NFIL3*) were shared across the three datasets (Figure 4(a)). The PPI results indicated a direct link between *CX3CR1*, *MYC,* and *TLR7* (Figure 4(b)). The functional similarity results showed a functional connection between *CX3CR1*, *MYC*, and *TLR7*, with *TLR7* occupying the most important position, followed by *CX3CR1* and *MYC* (Figure 4(c)).

### 3.5. Hub Gene Verification and Efficacy Evaluation

In the GSE55235 dataset, *CX3CR1* and *TLR7* levels increased, whereas *MYC* levels notably decreased, with a *P*-value <0.05 (Figures 5(a)–5(c)). In the validation datasets GSE51588 (Figures 5(d)–5(f)) and GSE55457 (Figures 5(g)–5(i)), the expression of the three genes was the same as that in the GSE51588 dataset, all of which were significant.

### 3.6. RT-qPCR Validation

The experimental results showed significantly increased expression of *CX3CR1* and *TLR7* in the OA group (Figures 6(a), 6(b)) and significantly decreased expression of *MYC* in the OA group (Figure 6(c)). The experimental results were in line with those obtained from the analysis of the three microarray datasets, demonstrating the reliability of our bioinformatics analysis results.

### 3.7. ROC Level Validation of Hub Genes

In the GSE55235 dataset, the true AUCs of CX3CR1 and TLR7 were greater than 0.9, and the true AUC of MYC was lesser than 0 (Figure 7(a)). In the validation datasets GSE51588 (Figure 7(b)) and GSE55457 (Figure 7(c)), the true AUCs of CX3CR1 and TLR7 were also greater than 0.9, and the true AUC of MYC was less than 0. CX3CR1 and TLR7 exhibited a strong ability to distinguish patients with OA from those without OA.

### 3.8. Immune Cell Infiltration

To deeply study the differential expression of immune components in OA and normal groups, the CIBERSORT algorithm was adopted for evaluating the relationship of OA phenotype with immune cell infiltration. The relative proportions of immune cell subtypes are shown in cumulative histograms (Figure 8(a)). The results showed that activated mast cells, CD4 naïve T cells, resting NK cells, and neutrophils accounted for a major proportion. The correlation heat map for 22 immune cell types (Figure 8(b)) showed a significant positive correlation between monocytes and eosinophils, a positive correlation between neutrophils and monocytes, and a negative association between resting and activated NK cells, and between eosinophils and resting dendritic cells. Besides, the violin plot regarding the difference in immune cell infiltration (Figure 8(c)) presented significantly more naive CD4 T cells, resting dendritic cells as well as activated NK cells compared to the normal control group.

### 3.9. Correlation Analysis of Hub Genes with Infiltration Degrees of Immune Cells

According to correlation analysis, *CX3CR1* exhibited a positive correlation with activated mast cells, NK cells, gamma delta T cells, and M1 macrophages. It was adversely related to resting CD4 memory T cells, activated CD4 memory T cells, neutrophils, and activated dendritic cells (Figure 9(a)). *TLR7* was in positive correlation with M2 macrophages, activated NK cells, M1 macrophages, gamma delta T cells, and resting dendritic cells. It was negatively related to activated dendritic cells and resting NK cells (Figure 9(b)). *MYC* was positively associated with resting CD4 memory T cells, eosinophils, neutrophils, activated dendritic cells, monocytes, and activated mast cells. It showed a negative correlation between activated mast cells and CD4 naive T cells (Figure 9(c)).

### 3.10. Drug Analysis Results

We used three mRNAs (CX3CR1, MYC, and TLR7) in the connectivity map (CMAP) database to predict potential drugs against OA. We found a variety of drugs for the treatment of OA, including Thapsigargin, Meteneprost, Naftifine, Trimethobenzamide, and Fludrocortisone (Table 2).

### 3.11. GSEA of Hub Gene

The GSEA was used to identify a complete list of gene sets enriched in *CX3CR1* (Figure 10(a)), *TLR7* (Figure 10(b)), and *MYC* (Figure 10(c)). Next, we selected immune-related gene sets from the complete list for further analysis. Six groups of genes were enriched in samples for CX3CR1, including “interferon-alpha response,” “allograft rejection,” “PI3K-AKT-MTOR signaling,” “inflammatory response,” “IL2-STAT5 signaling,” and “TNFA signaling via NF-KB” (Figure 11(a)). Similarly, “interferon-alpha response,” “allograft rejection,” “IL2-STAT5 signaling,” and “TNFA signaling via NF-KB” were enriched in TLR7-related samples (Figure 11(b)). Furthermore, the genomes of “interferon-alpha response,” “allograft rejection,” “inflammatory response,” “IL2-STAT5 signaling,” as well as “TNFA signaling via NF-KB” were enriched in MYC-related samples (Figure 11(c)).

## 4. Discussion

OA is the most common disease among the elderly and causes irreversible bone erosion and cartilage destruction [8]. Due to the lack of timely and efficient treatment, OA is bound to greatly influence the functions of a patient's joints. Although multiple diagnostic methods are available for OA, clinical outcomes have remained unsatisfactory. Furthermore, no drug therapy with convincing disease-modifying effects has been approved by regulatory agencies [9,10].

We used three datasets and found three biomarkers (CX3CR1, MYC, and TLR7), of which the AUC values of CX3CL1 and TLR7 were greater than 0.9 in all three datasets with good discrimination of OA capacity between patients of OA and healthy individuals. CX3CL1 is the only member of the CX3C chemokine class that has chemoattractant and adhesion molecule properties. CX3CL1 activates c-RAF, MEK, ERK, and NF*κ*B through the MMP-3 promoter of CX3CR1, thereby promoting the destruction of cartilage during OA [11]. CX3CR1 regulates the Wnt/*β*-catenin signaling, which consequently regulates the proliferation of chondrocytes and apoptosis in osteoarthropathy [12]. Toll-like receptor 7 (TLR7) is a single-stranded RNA pattern recognition receptor, and extracellular miR-21 released from synovial tissue mediates knee OA pain by activating the activation of TLR7 in surgical OA rat models [13]. TLR7 recognizes the microbes and endogenous RNAs, and nucleosides. Moreover, its aberrant activation has been implicated in numerous autoimmune diseases, including systemic lupus erythema (SLE) [14]. TLR7 detects viral RNA and can also be inappropriately activated by self-RNA, generating autoimmunity [15]. The *MYC* gene consists of three sub-branches, namely, *C-MYC*, *N-MYC*, and *L-MYC*, and is one of the most common runaway driver genes in human cancers [16]. The proto-oncogene *MYC* regulates several cellular processes, containing proliferation and metabolism. Keeping the homeostatic levels of *MYC* is vital for normal cell function; its overexpression is associated with several cancers. MYC stability can be regulated by phosphorylation, and phosphorylation signals at Thr58 degrade it, whereas Ser62 phosphorylation generates its stabilization and functional activation [17]. In addition, we used the CMAP database to identify multiple therapeutics targeting CX3CR1, MYC, and TLR7. However, their specific functions in OA and consequent side effects require further clinical studies. In the dataset GSE55235, the expression of CX3CR1 and TLR7 was significantly increased, and the expression of *MYC* was significantly reduced in patients with OA. The expression of the above three HUB genes was validated in the other two datasets. We found that the results of RT-qPCR validation for CX3CR1, MYC, and TLR7 were consistent with all three datasets, demonstrating the reliability of our results. Although the three studies used different gene expression analysis platforms and were conducted in highly distinct populations, the three gene levels remained unaffected. Furthermore, the above three genes were commonly expressed in different individuals. More investigations are needed to explore their levels and associated activities.

To further analyze the infiltration degree of immune cells within OA, a comprehensive evaluation of OA immune infiltration was performed using CIBERSORT. This study observed higher regulatory T cell and mast cell infiltration degrees, whereas reduced eosinophil, activated NK cell, and resting CD4^+^ T cell infiltration degrees, were associated with OA occurrence. A prior study reported relatively high mast cell infiltration in synovial tissues from OA cases and was associated with structural damage [18]. M2 cells are closely related to inflammation, such as having anti-inflammatory activity, and being regulated by squid type II collagen, thereby promoting cartilage repair under inflammatory conditions [19, 20]. Cartilage proteoglycans located in the G1 region can induce T cell responses and promote the degradation of cartilage in patients undergoing OA [21]. Apart from that, researchers have pointed out the abundance of regulatory T cells within OA, with their levels being related to the levels of inflammatory molecules [22]. As reported by Ezawa and colleagues, memory CD4^+^ T cells are universally accumulated in the case of local inflammatory response in joints, which are engaged in forming chronic OA [20]. Using *in vivo* experiments confirmed the important functions of neutrophils and NK cells in OA, and the interaction between them is stimulated via CXCL10/CXCR3 axis [23]. Based on this background and our findings, regulatory T cells, resting mast cells, activated NK cells, and resting CD4^+^ memory T cells exert a vital effect on OA pathogenesis, which will become a future research focus. Nevertheless, no research currently exists regarding eosinophils' effect on OA, requiring deep experimental analysis. Furthermore, our results revealed the infiltration degrees of 22 immune cell types within OA. Regulatory T cell and activated mast cell infiltration degrees were intricately associated with activated NK cell and resting CD4^+^ memory T cell infiltration. The infiltration degree of activated dendritic cells was in close correlation with eosinophilic infiltration. Again, specific mechanisms of the above-mentioned associations need the evidence of further experimental evidence.

An analysis of the association of CX3CR1, MYC, and TLR7 with immune cells revealed that CX3CR1 showed obvious positive relation to activated M1 macrophages, NK cells, gamma delta T cells, and activated mast cells, whereas activated CD4^+^ memory T cells, neutrophils, resting CD4^+^ memory T cell, and activated DCs were negatively correlated. TLR7 was significantly positively correlated with M1 macrophages, M2 macrophages, activated NK cells, resting dendritic cells, and gamma delta T cells, whereas notably adversely related to DCs and activated resting NK cells. MYC showed a significant positive relation with resting CD4^+^ memory T cells, eosinophils, neutrophils, activated DCs, monocytes, as well as activated mast cells, whereas it was markedly adversely linked with activated mast cells and CD4^+^ naive T cells. CX3CR1, MYC, and TLR7 are involved in immune processes. For instance, CX3CR1 is essential in airway inflammation and promotes the survival and maintenance of *T* helper cells in the inflamed lungs [24]. In addition, CX3CR1 modulates bacterial translocation, intestinal macrophage homeostasis, as well as colitis Th17 responses in mice [25]. CX3CR1 mediates the access of dendritic cells to the intestinal lumen and bacterial clearance. TLR7 induces anergic human CD4^+^ T cells [26]. Plasmacytoid dendritic cells (pDCs) sense the viral RNA through toll-like receptor 7 (TLR7), leading to the formation of self-adhesive pDC–pDC clusters and yield type I interferons. Besides, such cell adhesion can enhance the production of type I interferons [27]. Autophagy exerts a vital function in TLR7-mediated activation of B cells to induce SLE by delivering RNA ligands to endosomes, where innate immune receptors are located [28]. The MYC pathway not only determines cancer cell pathophysiology but also suppresses host immune responses [29]. MYC is known to regulate antitumor immune responses through CD47 and PD-L1. In addition, c-Myc is required for maintaining homeostasis and transient activation of regulatory T cells [16]. Studies have reported significant functions of NK cells and mast cells in OA. Because the polarization of M1 macrophages within synovium deteriorates OA [30], It can be speculated that CX3CR1 elevated the number of NK cells and naive CD4^+^ T cells or decreased the number of M1 macrophages, whereas MYC and TLR7 decreased the number of mast cells related to OA occurrence. These hypotheses need future studies to elucidate the complicated gene-immune cell interactions.

Furthermore, single-gene GSEA analysis revealed that “interferon-alpha response,” “allograft rejection,” “PI3K-AKT-MTOR signaling,” “inflammatory response,” “IL2-STAT5 signaling.” and “TNFA signaling via NFK-B” were involved in the OA immune process. Interferons can induce or exacerbate autoimmune diseases due to their immunomodulatory properties. For example, alpha-interferon can induce severe immune thrombocytopenia in those suffering from chronic hepatitis C. Moreover, probiotics that modulate the mTOR/PI3K/Akt signaling pathway can activate immune responses. PI3K and mTOR positively regulate the activation of immune cells of neutrophils and mast cells. In addition, T-cell receptors regulate the expression of Foxp3 through the PI3K/Akt/mTOR signaling network, thereby participating in immune processes. Dying neutrophils are known to produce anti-inflammatory effects by modulating surrounding cellular responses, especially macrophages that release inflammatory cytokines. Several cellular components of both adaptive and innate immune responses are present at the sites of tissue inflammation. Targeted delivery of IL2 to the tumor stroma can enhance the effects of immune checkpoint inhibitors by preferentially activating NK and CD8^+^ T cells. Furthermore, the tetramerization of STAT5 is important for cytokine responses and normal immune function, establishing its vital function *in vivo*. TTP53 GOF mutants up-regulate the expression of CC motif chemokine ligand 2 (CCL2) and TNFA via the NF*κ*B signaling pathway, thereby increasing microglia-and monocyte-derived immunity cell infiltration. The complex functions of CX3CR1, MYC, and TLR7 and these pathways in OA require elucidation.

Our study had certain limitations. First, the data used in the current work were acquired from public databases, with no way to validate the reliability of the data. Second, this study explored the association of OA markers with immune cells. Meanwhile, the reliability of this result in OA needs to be experimentally verified. Third, we did not deeply experimentally investigate the exact mechanism of the hub gene identified in OA.

## 5. Conclusion

Our study identified three hub genes, their relationship with the immune microenvironment, and certain functional biological pathways associated with immune response, inflammatory response, and cytokines related to O pathogenic mechanism. In addition, potential drugs for the treatment of OA were discovered. Although the obtained results offer new insights into OA genesis and progression, the exact molecular mechanism and functional pathway of HUB genes in OA still require to be deeply investigated.

## Figures and Tables

**Figure 1:** Analysis of EDGs (a): Volcano Plot of GSE55235 dataset:(b): Volcano Plot of GSE51588 dataset; (c): Volcano Plot of GSE55457 dataset; Up-regulated differentially expressed genes are indicated by red dots; down-regulated differentially expressed genes are indicated by blue dots; nonsignificant genes are indicated by gray dots. (d): Heat map of GSE55235 dataset; (e): Heat map of GSE51588 dataset (f): Heat map of GSE55457 dataset. Differential epigones that are highly expressed in the samples are marked in red, and differentially expressed genes that are low in the samples are indicated in blue.

**Figure 2:** Gsea (a): BP; (b): CC; (c): Mf; (d): Kegg.

**Figure 3:** GO Enrichment Analysis (a): BP; (b): CC; (c): MF; (d): KEGG. The size of the circle represents the number of genes; darker red means a smaller corrected *P* -value, and darker blue means a larger corrected *P* -value.

**Figure 4:** PPI network and Hub gene screening results. (a): Common up-regulated DGs of the three datasets; (b): Common down-regulated DGs of the three datasets; (c): PPI network of common DGs; (d): Function similarity analysis.

**Figure 5:** Expression levels of Hub genes (a): CX3CR1 expression levels in GSE55235 dataset; (b): MYC expression levels in GSE55235 dataset; (c): TLR7 expression levels in GSE55235 dataset; (d): CX3CR1 expression levels in GSE51588 dataset; (e): MYC expression levels in GSE51588 dataset; (f): TLR7 expression levels in GSE51588 dataset; (g): CX3CR1 expression levels in GSE55457 dataset; (h): MYC expression levels in GSE55457 dataset; (i): TLR7 expression levels in GSE55457 dataset.

**Figure 6:** Relative mRNA expression of EDGs (a): Relative mRNA expression of CX3CR1; (b): Relative mRNA expression of TLR7; (c): Relative mRNA expression of Myc.

**Figure 7:** ROC(Receiver Operating Characteristic) curves of Hub gene. (a): ROC curves of Hub gene in GSE55235; (b): ROC curves of Hub gene in GSE51588; (c): ROC curves of Hub gene in GSE55457; A larger ROC value represents a greater ability of the key gene to distinguish between OA and normal individuals.

**Figure 8:** Immune cell infiltration analysis (a): Immune cell percentage chart; (b): Correlation diagram between immune cells; (c): Expression of immune cells in OA group and Control group.

**Figure 9:** Correlation analysis of Hub genes and immune cells (a): Correlation analysis of CX3CR1 and immune cells; (b): Correlation analysis of MYC and immune cells; A Correlation analysis of TLR7 and immune cells; The magnitude of the absolute value of the correlation coefficient is indicated by the size of the circle. Larger *P* -values are indicated in dark purple, and smaller *P* -values are indicated in dark green.

**Figure 10:** GSEA analysis of HUB genes (a): Complete GSEA results for CX3CR1; (b): Complete GSEA results for MYC; (c): Complete GSEA results for TLR7; The number of genes is indicated by the size of the circle; smaller corrected *P*-values are indicated in dark red, and larger corrected *P*-values are indicated in dark blue.

**Figure 11:** Immune-related pathways of Hub genes (a): Immune-related GSEA results of CX3CR1 (b): Immune-related GSEA results of MYC (c): Immune-effective GSEA results of TLR7.

**Table 1:** | Primer sequences.

Gene	Primer (5′-3′)	
GAPDH	Forward	GACATGCCGCCTGGAGAAAC
GAPDH	Reverse	AGCCCAGGATGCCCTTTAGT
CX3CR1	Forward	CACCAAAGCCAGCACATAGGAGAG
CX3CR1	Reverse	GTCTGCGGATCTTGGACAAACAAATG
MYC	Forward	AGCAGCGACTCTGAAGAAGAACAAG
MYC	Reverse	GGATGACCCTGACTCGGACCTC
TLR7	Forward	GTATGCCACCGAATCTAACGACTCTC
TLR7	Reverse	GCCAATCTCGCAGGGACAGTTG

**Table 2:** mRNA was used to predict potential drugs for the treatment of OA.

Cmap name	Mean	*N*	Enrichment	*P*	Specificity	Non-null percent
Thapsigargin	−0.828	3	−0.977	0.00004	0.0129	100
Meteneprost	−0.781	4	−0.853	0.00088	0	100
Naftifine	−0.78	4	−0.884	0.0004	0	100
Trimethobenzamide	−0.702	5	−0.779	0.00096	0.0067	100
Fludrocortisone	−0.371	8	−0.648	0.00092	0.0493	50

## Data Availability

The data used to support this manuscript are included within this manuscript.

## Additional Points

1. In this study, we discovered that CX3CR1, MYC, and TLR7 could be used as a new diagnostic marker by bioinformatics methods and RT-qPCR, which provides a new direction for studying the pathogenesis of OA. 2. Using drug information from the CMAP database, we have identified multiple drugs that have effects on CX3CR1, MYC, and TLR7, providing potential therapeutic options for the treatment of OA. 3. Using GSEA, we have discovered multiple pathways involved in CX3CR1, MYC, and TLR7 in OA, further enriching our study of them.
